This article has been retracted.

# The response of nucleus pulposus cell senescence to static and dynamic compressions in a disc organ culture

**DOI:** 10.1042/BSR20180064

**Published:** 2018-03-09

**Authors:** Jianmin Shi, Lianglong Pang, Shouguo Jiao

**Affiliations:** 1 Department of Orthopaedics, Liaocheng People’s Hospital and Liaocheng Clinical School of Taishan Medical University, Liaocheng 252000, Shandong, China; 2 Department of Spine Surgery, Liaocheng People’s Hospital, Liaocheng 252000, Shandong, China; 3 Department of Orthopaedics, Yantai Yeda Hospital, Yantai 264006, Shandong, China

**Keywords:** compression, degeneration, nucleus pulposus, organ culture, senescence

## Abstract

Mechanical stimuli obviously affect disc nucleus pulposus (NP) biology. Previous studies have indicated that static compression exhibits detrimental effects on disc biology compared with dynamic compression. To study disc NP cell senescence under static compression and dynamic compression in a disc organ culture, porcine discs were cultured and subjected to compression (static compression: 0.4 MPa for 4 h once per day; dynamic compression: 0.4 MPa at a frequency of 1.0 Hz for 4 h once per day) for 7 days using a self-developed mechanically active bioreactor. The non-compressed discs were used as controls. Compared with the dynamic compression, static compression significantly promoted disc NP cell senescence, reflected by the increased senescence-associated β-galactosidase (SA-β-Gal) activity, senescence-associated heterochromatic foci (SAHF) formation and senescence markers expression, and the decreased telomerase (TE) activity and NP matrix biosynthesis. Static compression accelerates disc NP cell senescence compared with the dynamic compression in a disc organ culture. The present study provides that acceleration of NP cell senescence may be involved in previously reported static compression-mediated disc NP degenerative changes.

## Introduction

Low back pain (LBP) is a common and severe public health problem worldwide, which produces heavy economic burden and causes distress to patients [1]. LBP is closely correlated with intervertebral disc degeneration (IDD) [2]. Current treatments for IDD aim to relieve pain symptoms but not to interdict its pathogenesis [3]. Although several biological therapies are promising to retard mild to moderate disc degeneration [4,5], their clinical applications and efficacy need to be verified.

Apart from cell number, cellular morphology, and cell apoptosis, cellular senescence has been studied in the human disc recently [6–9]. These studies have reached a consensus that cellular senescence is positively correlated with the progressive degree of disc degeneration. Therefore, acceleration of disc cell senescence may be a potential approach for certain pathological risk factors aggravated disc degeneration.

Though the initial disc degeneration commonly occurs as a natural part of ageing process [10], increasing evidences indicate that inappropriate mechanical stimulation, an important external risk factor of IDD [11], can also contribute to disc cell senescence [12–14]. Under the physiological conditions, the disc is subjected to various kinds of mechanical loads [15]. During the past years, the static compression and dynamic compression have been well studied [16–18]. It is generally demonstrated that static compression imposes much more detrimental effects on disc biology compared with the dynamic compression [17]. However, whether disc cell senescence is responsible for the effect discrepancy between the static compression and dynamic compression is unknown.

Because the nucleus pulposus (NP) region first exhibits degenerative changes during disc degeneration [19], we mainly aimed to investigate the disc NP cell senescence under the static compression and dynamic compression in the present study. NP cell senescence was evaluated by several direct and indirect parameters, such as senescence-associated β-galactosidase (SA-β-Gal) activity, senescence-associated heterochromatic foci (SAHF), telomerase (TE) activity, senescence markers expression (p16 and p53), and matrix homeostatic phenotype.

## Materials and methods

### Ethical statement

All animal experiments were performed according to the guidelines of the Ethics Committee at Liaocheng People’s Hospital and Liaocheng Clinical School of Taishan Medical University (SLJS (LU) 2009-0014).

### Disc harvest and bioreactor culture

Fifteen healthy pigs (3–4 months old and 12–13) were used in the present study. The intact discs (T11-L5) were harvested with cartilage end plates under sterile conditions as described previously [20]. After washing with PBS, the anterior-posterior and lateral widths were measured to calculate the disc area (Area ≈ π(WapWlat)/4, where the Wap and Wlat are the anterior-posterior and lateral widths, respectively) [21]. Then, the compressive magnitude in the form of pressure (MPa) was converted into the compressive magnitude in the form of newtonian (N). All discs were cultured and compressed (static compression: 0.4 MPa for 4 h once per day; dynamic compression: 0.4 MPa at a frequency of 1.0 Hz for 4 h once per day) for 7 days using a mechanically active perfusion bioreactor. The control discs were not compressed. To decrease interference of compressive magnitude on NP cell senescence, the magnitude of 0.4 MPa was designed because it is a relatively healthy compressive magnitude [22], which approximately equals the intradisc pressure when a person is in the upright position [23]. The discs were kept in sterile DMEM/F12 culture (HyClone, U.S.A.) containing 10% (v/v) FBS (Gibco, U.S.A.), and 1% (v/v) penicillin-streptomycin (Gibco, U.S.A.). To avoid the interference caused by differences at vertebral level, each experiment was performed on the same three discs (L1/2, L2/3, and L3/4) from different animals as described previously [24].

### SA-β-Gal staining assay

After compression, the central NP tissue was immediately isolated by digestion with 0.25% trypsin (HyClone, U.S.A.) and 0.25% Type I collagenase (Sigma, U.S.A.). Then, NP cell pellets were suspended for 4–5 h to allow cell attachment. SA-β-Gal staining was carried out using a Senescence β-Galactosidase Staining Kit (Beyotime, China). Finally, NP cells were observed under a light microscope (Olympus BX51, Japan). SA-β-Gal activity was reflected as the percentage of staining-positive NP cells to total NP cells.

### SAHF formation

After culture, discs were fixed with 4% paraformaldehyde, decalcified with 10% EDTA, and embedded in paraffin. Subsequently, 5-μm-thick cross-sections were stained with DAPI solution (Beyotime, China). The positive stain was recorded using a laser scanning confocal microscope (Zeiss, LSM780, Germany). The percentage of SAHF-positive NP cells was calculated using ImagePro Plus software (version 5.1, Media Cybernetics, Inc.).

### TE activity

Briefly, after the central disc NP tissue was isolated and NP cell pellets were collected as described above, NP cell pellets were lysed and centrifuged to obtain supernatant. Then, a TE ELISA kit (Mlbio, China) was used to measure TE activity (IU/l).

### Real-time PCR analysis

Briefly, total RNA was extracted from the isolated central NP tissue using TRIzol reagent (Invitrogen, U.S.A.). RNA quality and concentration were analyzed using the Nanodrop ND-1000 Spectrophotometer (Nanodrop Technologies). Then, 1 μg of RNA was reverse-transcribed into cDNA product. Finally, real-time PCR was performed in triplicate on a reaction mixture containing cDNA, SYBR Green Mix (TOYOBO, Japan) and primers (Table 1). The reaction conditions of thermal cycling were: 3 min at 92°C, followed by 30 amplification cycles of 20 s at 95°C, 10 s at 57°C, and 15 s at 72°C. GAPDH was used as an internal reference. The relative expression was calculated using the method of 2^―ΔΔ*C*^_t_.

**Table 1:** Primers of target genes

Gene	Accession number	Forward (5′–3′)	Reverse (5′–3′)
*GAPDH*	NM_001206359.1	ACCTCCACTACATGGTCTACA	ATGACAAGCTTCCCGTTCTC
*Aggrecan*	NM_001164652.1	CGTGGTCCAGCACTTCTAAA	AGTCCACTGAGATCCTCTACTC
*Collagen II*	XM_001925959.4	CCGGGTGAACGTGGAGAGACTG	CGCCCCCACAGTGCCCTC
*P16*	XM_013993499.1	TGCAGTTGCCTACCTCTGAA	CGAATCCGCACAGTAATCAA
*P53*	NM_213824.3	CCTTAAGATCCGTGGGCGT	GCTAGCAGTTTGGGCTTTCC

### Immunohistochemistry staining

Briefly, 5-μm-thick disc cross-sections were processed through deparaffination, inactivation of endogenous peroxidase, and enzyme antigen retrieval. Then, disc sections were washed with PBS and incubated with 5% BSA for 12 min at room temperature. Thereafter, sections were incubated at 4°C overnight with primary antibodies (aggrecan: Novus, NB120-11570, diluted 1:200; collagen II: Abcam, ab34712, diluted 1:200). After washing with PBS for two to three times, sections were incubated at 37°C for 2 h with corresponding HRP-conjugated secondary antibodies (goat anti-mouse IgG and goat anti-rabbit IgG, ZSGB-BIO, China, diluted 1:300). Finally, sections were washed, color-developed with diaminobenzidine (DAB) and counterstained with Hematoxylin. Randomly selected images were recorded using a light microscope (Olympus BX51). The staining intensity was quantitated using the ImagePro Plus software (version 5.1, Media Cybernetics, Inc.).

### Western blotting assay

Briefly, total protein was extracted from the isolated NP samples using the RIPA lysis solution (Beyotime, China), and then protein concentration was measured using a Nanodrop ND-1000 Spectrophotometer (Nanodrop Technologies). Thereafter, equal amount of protein samples in each group was resolved by SDS/PAGE and transferred on to the PVDF membrane. After blocking with 5% BSA for 2 h at room temperature, the PVDF membrane was incubated with the primary antibodies (p53: Biosource, #MBS8242548; p16: Santa Cruz Biotechnology, sc-28260; GAPDH: Abcam, ab8245) overnight at 4°C. Next, the membranes were incubated at 37°C for 2 h with corresponding HRP-conjugated secondary antibodies (goat anti-mouse IgG and goat anti-rabbit IgG, ZSGB-BIO, China, diluted 1:4000). Protein bands were developed using the ECL method (Thermo, U.S.A.). After the gray value of protein bands were measured using the ImageJ software (National Institutes of Health, U.S.A.), the ratio of the density of p16 or p53 to the density of GAPDH was calculated.

### Biochemical content measurement

Briefly, NP tissue samples were immediately isolated as described after culture. Then, glycosaminoglycan (GAG) content was measured using the dimethyl methylene blue (DMMB) method as previously described [25], and the hydroxyproline (HYP) content was measured using an HYP measurement detection kit (Nanjing Jiancheng, China) according to the manufacturer’s instructions.

### Statistics

All numerical data were expressed as the means ± S.D. Each experiment was performed at least in triplicate. The statistical differences amongst these groups were analyzed using one-way ANOVA and the LSD test as a post hoc test. A *P*-value <0.05 was considered statistically significant.

## Results

### SA-β-Gal activity

Compared with the control group, static compression increased SA-β-Gal activity of NP cells, whereas dynamic compression decreased SA-β-Gal activity of NP cells. Additionally, SA-β-Gal activity in the static compression group was significantly higher than in the dynamic compression group (Figure 1).

**Figure 1:** SA-β-Gal staining of NP cells from porcine discs subjected to static and dynamic compression The data are expressed as the means ± S.D., *n*=3. ^#^: Indicates a significant difference compared with the control group. *: Indicates a significant difference between two groups (*P*<0.05).

### SAHF observation

Results showed that the percentage of SAHF-positive NP cells in the static compression group was higher whereas it was lower in the dynamic compression group than that in the control group. Additionally, the percentage of SAHF-positive NP cells in the static compression group was significantly increased compared with that in the dynamic compression group (Figure 2).

**Figure 2:** Quantitation of cell fraction in each cell cycle phase (G_0_/G_1_, S, and G_2_/M) in NP cells from porcine discs subjected to static and dynamic compression (*n*=3)

### TE activity

TE activity results showed that it was decreased in the static compression group and increased in the dynamic compression group compared with the control group. However, the TE activity in the static compression group was significantly lower than that in the dynamic compression group (Figure 3).

**Figure 3:** TE activity in NP cells from porcine discs subjected to static and dynamic compression The data are expressed as the means ± S.D., *n*=3. ^#^: Indicates a significant difference compared with the control group. *: Indicates a significant difference between two groups (*P*<0.05).

### Senescence markers expression

Real-time PCR analysis showed that gene expression of senescence markers (p16 and p53) was up-regulated in the static compression group, whereas down-regulated in the dynamic compression group compared with the control group. Additionally, they were significantly decreased in the dynamic compression group compared with the static compression group (Figure 4A). Similarly, Western blotting assay showed that protein expression of these senescence markers (p16 and p53) exhibited a similar trend to their gene expression amongst these groups (Figure 4B).

**Figure 4:** Analysis of senescence markers (p16, p21, and p53) expression in NP cells of porcine discs subjected to static and dynamic compression (**A**) Real-time PCR analysis of *p16* and *p53* mRNA expression. (**B**) Western blot analysis of p16 and p53 protein expression. The data are expressed as the means ± S.D., *n*=3. ^#^: Indicates a significant difference compared with the control group, respectively. *: Indicates a significant difference between two groups (*P*<0.05).

### Matrix macromolecules expression

Results showed that gene expression of NP matrix macromolecules (aggrecan and collagen II) was down-regulated in the static compression group and up-regulated in the dynamic compression group compared with the control group, but they were significantly decreased in the static compression group compared with the dynamic compression group (Figure 5A). In-line with this, immunohistochemical staining showed that protein deposition in these NP matrix macromolecules presented a similar trend to their gene expression profile amongst these groups (Figure 5B).

**Figure 5:** Matrix homeostatic phenotype in NP cells of porcine discs subjected to static and dynamic compression (**A**) Real-time PCR analysis of matrix macromolecules (aggrecan and collagen II). (**B**) Immunohistochemistry analysis of matrix macromolecules (aggrecan and collagen II). The data are expressed as the means ± SD, *n*=3. ^#^: Indicates a significant difference compared with the control group. *: Indicates a significant difference between two groups (*P*<0.05).

### Matrix biochemical content

GAG and HYP content analysis showed that they were decreased in the static compression group and increased in the dynamic compression group compared with the control group. However, both GAG content and HYP content in the static compression group were significantly decreased compared with the dynamic compression group (Figure 6).

**Figure 6:** Biochemical content measurement Analysis of GAG content (**A**) and HYP content (**B**) in NP cells of porcine discs subjected to static and dynamic compression. The data are expressed as the means ± S.D., *n*=3. ^#^: Indicates a significant difference compared with the control group. *: Indicates a significant difference between two groups (*P*<0.05).

## Discussion

Mechanical stimuli can cause diverse effects on disc cells, depending on the loading type, magnitude, duration, and disc cell origination [15]. Under physiological conditions, the disc experiences various physical stimuli, including compression, tensile, shear stress, and hydrostatic pressure [26]. In most cases, the disc NP is predicted to mainly experience axial compression [26]. Previous studies indicate that static compression has detrimental effects on disc cell biology compared with the dynamic compression [17]. However, the potential mechanism is not fully investigated. Acceleration of disc cell senescence is potentially responsible for mechanical load-induced disc degenerative changes [12–14]. These studies demonstrated that static compression significantly promoted disc NP cell senescence compared with the dynamic compression in a disc organ culture. The present study provides a possible mechanism underlying the different effects on disc NP cell biology between the static compression and dynamic compression.

Until now, several classical parameters have been used to evaluate cellular senescence, such as SA-β-Gal activity, SAHF formation, and TE activity; and senescent cells often have increased SA-β-Gal activity, promoted SAHF formation, and decreased TE activity [27–29]. In the present study, we found that static compression significantly increased SA-β-Gal activity, promoted SAHF formation, and decreased TE activity in disc NP cells compared with the dynamic compression, indicating that static compression can accelerate disc NP cell senescence compared with the dynamic compression. In light of the previously reported negative effects of static compression on disc NP cell viability and NP matrix biosynthesis compared with the dynamic compression, we deduced that the acceleration of disc NP cell senescence may be the possible reason for this discrepancy in the response of disc NP cells to static and dynamic compression.

According to previous opinion, there are two mechanisms mediating cellular senescence. One is the replicative senescence (RS) and the other is stress-induced premature senescence (SIPS) [12]. The telomere-based p53-p21-pRB pathway and the stress-based p16-pRB pathway are involved in these two mechanisms, respectively [12]. Previously, disc NP cell senescence has been identified and is suggested to be positively correlated with disc degeneration advancing [6–9]. In this study, we found that static compression significantly up-regulated expression of senescence markers (p16 and p53) of NP cells both at gene and protein levels, again indicating that static compression can promote disc NP cell senescence compared with the dynamic compression, and that both the RS and SIPS may simultaneously participate in the static compression-induced disc NP cell senescence. Similar to this to some extent, a previous study has reported that expression of either p16 or p53 or both of them are simultaneously increased in the degenerative disc tissue [30]. Collectively, it can be speculated that attenuating disc NP cell senescence may be promising to retard static compression-induced disc NP degeneration.

Matrix homeostatic phenotype is an indirect parameter to evaluate cellular senescence since senescent cells often exhibit catabolism-like matrix metabolism [31]. Aggrecan and collagen II are two main macromolecules within the disc NP region [32]. Our results showed that static compression significantly decreased gene expression and their protein deposition in disc NP cells compared with dynamic compression; similarly, NP matrix biochemical (GAG and HYP) content in the static compression group was obviously lower than in the dynamic compression group. These results are consistent with a previous study which reflects that static compression causes a catabolic matrix metabolism compared with the dynamic compression [17]. On the other hand, this also again suggests that static compression facilitates senescence-like phenotype in disc NP cells compared with the dynamic compression.

Though the present study reported some important information, it has several inevitable limitations. First, because notochordal cells almost disappeared within the adult human disc NP region, the existence of notochordal cells within the immature porcine disc NP tissue may limit present study’s stringency in imitating the mechanobiology of the adult disc [33]. Second, though we demonstrate that static compression can obviously promote disc NP cell senescence compared with dynamic compression, the potential signaling transduction is not investigated. Previous studies have demonstrated that MAPK pathways and Wnt pathways are activated under mechanical stimulation. However, this needs to be further studied in the future.

In conclusion, static compression aggravates disc NP cell senescence compared with the dynamic compression in a disc organ culture. The present study indirectly provides a possible mechanism underlying the previously reported negative effects of static compression on disc NP cell biology.

## Abbreviations

DMEM/F12: Dulbeco’s Modified Eagle Media:Nutrient Mixture F-12
GAG: glycosaminoglycan
GAPDH: glyceraldehyde-3-phosphate dehydrogenase
HRP: horse radish peroxidase
HYP: hydroxyproline
IDD: intervertebral disc degeneration
LBP: low back pain
MAPK: mitogen-activated protein kinase
NP: nucleus pulposus
RS: replicative senescence
SAHF: senescence-associated heterochromatic foci
SA-β-Gal: senescence-associated β-galactosidase
SIPS: stress-induced premature senescence
TE: telomerase
